# Expression and Significance of D-Dimer and Fibrinogen in Hyperfibrinolysis of Elderly Patients with Bleeding after BPH Operation

**DOI:** 10.1155/2022/9387484

**Published:** 2022-07-20

**Authors:** Zhaoyue Liu, Huifang Yan, Shanshan Jin, Jingzhang Wu, Zhanwu Zhang, Qian Yu

**Affiliations:** ^1^Department of Urology, Hengshui People's Hospital, Hengshui, China; ^2^Department of Pediatrics, Hengshui People's Hospital, Hengshui, China

## Abstract

**Objective:**

To explore the expression level and diagnostic efficacy of plasma D-dimer (DD) and fibrinogen (FIB) in hyperfibrinolysis of elderly patients with bleeding after benign prostatic hyperplasia (BPH) surgery.

**Methods:**

70 elderly BPH patients with postoperative hemorrhage and hyperfibrinolysis in our hospital were included into the observation group, and 75 elderly BPH patients with postoperative hemorrhage without hyperfibrinolysis were included into the control group. The serum levels of DD and FIB in the two groups of patients were compared, and the correlation of DD and FIB with clinical features and the diagnostic value of DD and FIB.

**Results:**

Elderly BPH patients with hyperfibrinolysis showed significantly higher levels of DD and FIB than those without hyperfibrinolysis (*P* < 0.01). The increase in DD and the decrease of FIB were significantly correlated with the prolonged hospital stay and intensive care unit (ICU) monitoring (*P* < 0.05). The combination of DD and FIB showed high diagnostic value for postoperative hemorrhage with hyperfibrinolysis (AUC = 0.998).

**Conclusion:**

The combination of plasma DD and FIB effectively and accurately diagnoses postoperative hemorrhage with hyperfibrinolysis. High levels of DD and FIB indicate prolonged hospital stay and postoperative ICU monitoring of elderly BPH patients with hyperfibrinolysis.

## 1. Introduction

Benign prostatic hyperplasia (BPH) is the main cause of dysuria in elderly males [1]. It is the result of hyperplasia of epithelial and fibromuscular tissue in the transitional zone of the prostate and in the periurethral region. At present, transurethral resection of prostate (TURP) is the standard treatment protocol for BPH, and suprapubic enucleation procedures have been criticized due to relatively high transfusion and revision rates and and prolonged hospital stay. Hemorrhage is a common complication after TURP, with an incidence of about 12% [2, 3]. Bleeding after prostatectomy may lead to hyperfibrinolysis. The change of D-dimer (DD) is of great value in the diagnosis and evaluation of sepsis and deep vein thrombosis. Fibrinogen (FIB) is an important factor to evaluate coagulation function and reflects the degree of inflammatory response [4, 5]. Traditional Chinese medicine believed that BPH site of stagnation is in the bladder, which is related to the kidney, liver, spleen, and lung, and blood stasis and damp-heat are the pathological basis of its pathogenesis. Bladder gasification dysfunction is the direct cause of its pathogenesis. The purpose of this study was to explore the expression level and diagnostic value of DD and FIB in elderly BPH patients with postoperative hemorrhage and hyperfibrinolysis and to explain the correlation of the functional state of coagulation and fibrinolysis system with the clinical characteristics of elderly BPH patients with postoperative hemorrhage and hyperfibrinolysis.

## 2. Materials and Methods

### 2.1. General Information

70 elderly BPH patients with postoperative hemorrhage and hyperfibrinolysis in our hospital from June 2018 to June 2020 were included in the observation group, and 75 elderly BPH patients with postoperative hemorrhage without hyperfibrinolysis were included in the control group.

Inclusion criteria [6]: patients who meet the diagnostic criteria in the guidelines for diagnosis and treatment of benign prostatic hyperplasia and are confirmed by ultrasound examination, aged over 60 years, and with complete clinical data were included.

Exclusion criteria: patients with bladder cancer, prostate cancer, and other malignant tumors, with abnormal consciousness after the operation, who received drugs affecting anticoagulation orally one week before the operation, with abnormal coagulation function before the operation, and with neurological dysfunction were excluded.

There were 70 cases of hyperfibrinolysis after prostatectomy. The age ranged from 62 to 79 (65.8) years old. There were 56 cases of grade II prostatic hyperplasia and 14 cases of grade III and II prostatic hyperplasia with preoperative rectal indications. B-ultrasound indicated 80–490 ml of residual urine. The average prostate-specific antigen (PSA) was 2.4 *μ*g/L, the maximum urine flow rate measured by urodynamics was 4.0–11.5 ml/s, the International Prostate Symptom Score (IPSS) was 20–35 points, and the quality of life score ranged from 2 to 6 points.

There were 75 cases of bleeding after prostatectomy without hyperfibrinolysis. The age ranged from 63 to 85 (67.9) years old. There were 50 cases of grade II prostatic hyperplasia and 25 cases of grade III and II prostatic hyperplasia with preoperative rectal indications. B-ultrasound indicated 75∼490 ml of residual urine. The maximum urine flow rate measured by urodynamics was 4.2∼11.3 ml/s, the average PSA was 2.5 *μ*g/L, the IPSS was 20–35 points, and the quality of life score was 2–6 points. There was no significant difference in age, prostate volume, residual urine volume, urinary flow rate, and IPSS score between the two groups (*P* > 0.05).

### 2.2. Research Methods

The clinical data of the patients such as age, postoperative bleeding volume, and hospital stay was collected. According to the above clinical characteristics, the difference between DD and FIB expression in the two groups was analyzed, and DD and FIB before treatment were collected for comparative analysis.

### 2.3. Index Detection

4 ml of morning fasting venous blood was collected on the next day after the operation. 2 ml was placed in an anticoagulant tube containing ethylenediaminetetraacetic acid (EDTA) and detected by the XN350 automated hematology analyzer (Sysmex, Japan). The remaining 2 ml of blood were injected into a sodium citrate anticoagulation tube and centrifuged at 3500 r/min for 10 min. The supernatant was collected for FIB and DD detection using the CS5100 automatic blood coagulation instrument (Sysmex, Japan).

### 2.4. Statistical Analysis

SPSS 25.0 was used for data analyses. The data of the two groups of samples were tested by *t*-test. Multivariate logistic regression was performed, and ROC curve was plotted. The diagnostic performance of the observed indicators was evaluated, and the area under the curve (AUC) was calculated. The best diagnostic efficiency was obtained based on the Yoden index (YI).

## 3. Results

### 3.1. Expressions of DD and FIB

Elderly BPH patients with postoperative hemorrhage and hyperfibrinolysis showed significantly higher expressions of DD and FIB versus those without hyperfibrinolysis (*P* < 0.05, Table 1).

### 3.2. Correlation Analysis of DD, FIB, and Clinical Characteristics in Elderly BPH Patients with Postoperative Hemorrhage and Hyperfibrinolysis

In elderly BPH patients with hyperfibrinolysis, the plasma DD concentration was associated with a hospital stay and ICU monitoring after the operation (*P* < 0.05) (Table 2). Plasma FIB was associated with systemic diseases, tracheotomy, hospital stay, and ICU monitoring after the operation (*P* < 0.05) (Table 3).

### 3.3. Regression Analysis

Logistic regression analysis showed that hospital stay (>10 days) and postoperative ICU monitoring of patients with high plasma DD were 6.5 times (95% CI: 1.687∼25.631) and 5.7 times (95% CI: 1.929∼16.381) higher than patients with low plasma DD. The hospital stay (>10 days) and postoperative ICU monitoring of patients with low levels of FIB were 3.6 times (95% CI: 1.318∼12.071) and 22 times (95% CI: 5.297∼83.975) higher than patients with high levels of FIB, and the probability of tracheotomy during the operation was 7.9 times higher than that of patients with high levels of FIB (95% CI: 2.781∼22.064). Elevated DD and decreased FIB in plasma are the risk factors affecting the length of hospital stay and ICU monitoring after the operation (Tables 4 and 5).

### 3.4. Efficacy Evaluation

The diagnostic efficacy of the combined detection of plasma DD and FIB is higher than that of single detection of either DD or FIB (Table 6).

## 4. Discussion

BPH is a common disease in urology, with a high prevalence in middle-aged and elderly males. Its clinical manifestations include urgent urination, frequent urination, residual urine, and dysuria [7,8]. The pathogenesis of BPH is that the increase in mitosis leads to an increase in the volume of parenchymal cells and tissues, resulting in greater urethral resistance and symptoms such as urinary urgency, frequency, and difficulty in urination [9]. Surgical resection of prostate tissue is the mainstay of treatment for BPH. Wounds after prostatectomy usually require 2 to 3 months to be covered by a new urethral mucosa, while complete wound epithelialization requires about 6 months. Related studies suggested that systemic factors were mostly related to long-term bleeding [10]. Therefore, a detailed medical history prior to surgery is indicated, and systemic diseases, especially hypertension, diabetes mellitus, and heart disease, require active and effective treatment.

Hyperfibrinolysis includes primary and secondary hyperfibrinolysis. The primary one is defined as the condition that plasminogen is activated to plasmin, or plasmin inhibitor is reduced, causing hyperplasminemia and then degrading fibrinogen and intermediating other plasma coagulation factors, resulting in a hypocoagulable state dominated by hypofibrinogenemia. Secondary hyperfibrinolysis is induced by enhanced coagulation mechanisms in the early stage of the disease with massive fibrin production, thereby causing hyperfibrinolysis [11]. Plasma D-dimer is the specific product of fibrin degradation. Measurement of plasma D-dimer facilitates the determination of the presence or absence of fibrin production and thus provides a basis for distinguishing primary from secondary fibrinolysis. This study showed that patients were diagnosed with secondary fibrinolysis with a D-dimer >565 *μ*g/L. FIB, also known as coagulation factor I, is a crucial index reflecting acute inflammation [12], and its concentration increases during severe infection, thrombosis, and vascular injury. In the presence of a series of coagulation factors, FIB forms cross-linked fibrin, and one of the characteristic products of degradation is DD, which is the main index of secondary hyperfibrinolysis [13]. DD was used to exclude the clinical diagnosis of deep vein thrombosis and pulmonary embolism, and FIB was used to assess coagulation function and prethrombotic state. Some studies have suggested that the expression of DD and FIB in the plasma of elderly BPH patients with hyperfibrinolysis after postoperative hemorrhage was abnormal and gradually recovered after effective treatment, but there was no research combining the clinical characteristics and diagnostic efficacy of the disease [14]. Hyperfibrinolysis promoted by bleeding after prostatectomy is secondary hyperfibrinolysis. Routine preoperative screening for coagulation effectively excludes primary hyperfibrinolysis, which reduces the risk of surgery and avoids postoperative bleeding of the prostate due to primary diseases [15]. Rapid and massive bleeding after prostatectomy causes massive blood clots in the bladder, which will induce secondary hyperfibrinolysis [16].

To our knowledge, FIB is a plasma glycoprotein synthesized by the liver and belongs to the acute phase protein, which is converted into fibrin monomer under the action of thrombin and then cross-linked into fibrin. It is the main component of thrombus and participates in the process of coagulation; DD is formed by cross-linked fibrin under the action of plasmin, which can reflect both the activity of thrombin and plasmin in vivo and can be used as a marker for the enhancement of secondary fibrinolytic activity, especially in the coexistence of thrombolysis and formation. It is important in the presence of activated thrombus. This study found that DD and FIB exhibited high specificity and sensitivity in the diagnosis of hyperfibrinolysis caused by postoperative hemorrhage in elderly BPH patients. The increase in DD was closely related to the prolonged hospital stay and postoperative ICU monitoring, while the decrease in FIB was related to systemic diseases and tracheotomy. FIB and DD show certain predictive value for early diagnosis of postoperative hemorrhage and fibrinolysis in elderly patients with BPH, and the combined prediction of FIB and DD improves the diagnostic predictive value of postoperative hemorrhage and fibrinolysis. Massive bleeding after BPH will induce massive blood clots in the bladder and secondary hyperfibrinolysis. because the reason may be that blood clots require absorption of substantial amounts of FIB and coagulation factors, and blood clots may cause hyperfibrinolysis during decomposition. Therefore, the color and flow rate of bladder irrigation fluid should be closely observed after the operation. If the color is persistently deep red or blood clots fill the bladder, the blood clots in the bladder should be removed timely to reduce the adsorption of blood clots to coagulation factors and fibrinogen.

Previously, traditional Chinese medicine treatments have yielded favorable results. For instance sitz bath (drug composition: leech, Hedyotis diffusa, cinnamon, cork, psyllium, triangular, curcuma, rhubarb, safflower, lychee seed, decoct and extract the juice in a special basin, the water temperature is 38∼42°C, sitz bath 20–40 min) combined with local massage therapy was used for BPH and produced a pronounced efficacy with a higher safety profile. Armed with the prior results, traditional Chinese medicine treatments should be promoted in the future.

To sum up, the combination of DD and FIB in plasma effectively and accurately diagnoses hyperfibrinolysis caused by postoperative hemorrhage. High levels of DD and FIB are important reference indicators for prolonged hospital and ICU monitoring of elderly BPH patients with postoperative hemorrhage and hyperfibrinolysis. Enhanced monitoring of DD and FIB before and after treatment facilitates the development of a comprehensive and effective treatment plan and improves clinical efficacy.

## Figures and Tables

**Table 1:** Comparison of plasma DD and FIB between two groups.

Group	N	DD(*μ*g/L)	FIB(g/L)
Observation group	75	567.32 ± 89.56	2.62 ± 0.95
Control group	70	376.51 ± 91.27	5.89 ± 0.68
T		5.354	6.734
P		0.001	≤0.001

**Table 2:** Relationship between plasma DD and clinical characteristics of elderly BPH patients with postoperative hemorrhage and hyperfibrinolysis.

Clinical features	n	Concentration (*μ*g/L)	t	*P*
Systemic diseases			1.528	0.103
Yes	33	578.29 ± 88.63		
No	37	565.71 ± 88.26		

Blood loss after operation			2.782	0.068
<500 ml	43	592.14 ± 86.55		
≥500 ml	27	581.35 ± 87.19		

Tracheotomy			1.626	0.098
Yes	30	592.61 ± 85.72		
No	40	578.19 ± 86.41		

Hospitalization stay (d)			3.957	0.004
≤10	25	557.25 ± 84.25		
>10	45	635.28 ± 86.83		

Postoperative ICU			2.871	0.016
Yes	23	629.15 ± 85.31		
No	47	551.92 ± 86.25		

**Table 3:** Relationship between plasma FIB and clinical characteristics of elderly BPH patients with postoperative hemorrhage and hyperfibrinolysis.

Clinical features	n	Concentration (*μ*g/L)	t	*P*
Systemic diseases			4.125	0.003
Yes	36	2.31 ± 0.85		
No	34	3.09 ± 0.63		

Blood loss after operation			1.431	0.257
<500 ml	46	2.55 ± 0.66		
≥500 ml	24	2.69 ± 0.72		

Tracheotomy			4.625	≤0.001
Yes	32	2.26 ± 0.74		
No	38	2.98 ± 0.65		

Hospitalization stay (d)			2.971	0.015
≤10	24	2.98 ± 0.65		
>10	46	2.25 ± 0.69		

Postoperative ICU			5.865	≤0.001
Yes	22	2.37 ± 0.73		
No	48	3.01 ± 0.84		

**Table 4:** Logistic regression analysis of plasma DD and clinical characteristics of elderly BPH patients with postoperative hemorrhage and hyperfibrinolysis.

Indicators	B	S.E	Wald	OR	95%CI		*P* Value
					Upper limit	Lower limit	
Hospitalization stay	1.851	0.679	8.347	6.513	1.687∼25.631		0.005
Postoperative ICU	1.706	0.381	14.367	5.703	1.929∼16.381		0.001

**Table 5:** Logistic regression analysis of plasma FBI and clinical characteristics of elderly BPH patients with postoperative hemorrhage and hyperfibrinolysis.

Indicators	B	S.E	Wald	OR	95%CI		*P* Value
					Upper limit	Lower limit	
Hospitalization stay	1.345	0.512	5.927	3.639	1.318∼12.071		0.012
Postoperative ICU	3.108	0.698	16.961	22.041	5.297∼83.975		0.001
Systemic diseases	−0.053	0.228	0.053	0.918			0.768
Tracheotomy	2.072	0.517	14.376	7.901	2.781∼22.064		0.008

**Table 6:** Diagnostic efficacy of plasma DD and FIB in elderly BPH patients with postoperative hemorrhage and hyperfibrinolysis.

Indicators	AUC	Critical value	Sensitivity	Specificity	YI
DD	0.917	565	82.3	95.7	0.772
FIB	0.929	2.36	95.3	96.8	0.958
DD + FIB	0.998		98.5	100	0.986

## Data Availability

No data were used to support this study.
